# Music Classification Method Using Big Data Feature Extraction and Neural Networks

This article has been retracted.

**DOI:** 10.1155/2022/5749359

**Published:** 2022-07-30

**Authors:** Xiabin Li, Jin Li

**Affiliations:** Lingnan Normal University, Zhanjiang 524048, China

## Abstract

From the cassette era to the CD era to the digital music era, the quantity of music has grown rapidly. People cannot easily search for the desired music without classifying enormous music resources and developing a successful music retrieval system. By examining users' historical listening patterns for personalised recommendations, the music recommendation algorithm can lessen message fatigue for users and enhance user experience. Relying on manual labelling is how traditional music is classified. It would be inefficient and unrealistic to attempt to classify music using manual labelling in the age of big data. Feature extraction and neural networks are the tools employed in this paper. The model's parameters can be trained using conventional gradient descent techniques, and the model's trained convolution neural network can learn the image's features and finish the extraction and classification of the features. This algorithm is 12 percent superior to the conventional algorithm, according to the research in this paper. It has strong ability and is appropriate for widespread implementation with the same number of iterations.

## 1. Introduction

Deep learning has advanced quickly as a result of the current rapid development of computing technology, which has improved computers' ability to process data. Artificial intelligence has made significant advances in recent years in the areas of speech recognition, unmanned driving, video analysis, etc. These advancements have been put to practical use and have produced positive outcomes. Due to the wide variety of musical genres and listening preferences among the audience, many people enjoy listening to music [1]. It will be much easier for people to find songs if the music library can be categorised, allowing listeners to selectively listen to their favourite songs through music classification labels. The development and use of music recommendation algorithms are only intended to address this issue. According to the user's behaviour message and the characteristics of the music data, the music recommendation algorithm predicts the user's behaviour preference and actively pushes music to users. More music is available for people to choose from, but it is challenging for people to find the music they are looking for in the vast music resources, which results in low retrieval efficiency [2]. Establish a great music index system after reasonably classifying the vast music resources to help people find the music they want more easily, increase the effectiveness of music retrieval, and then enhance how people search for and enjoy music. This will help people get the most enjoyment possible from music. In a music retrieval system, the calibre of music classification is obvious [3]. Numerous practical issues have been resolved with the development of the music recommendation algorithm, and its technical path has changed in recent years from the initial recommendation based on users' behavioural preferences to the association recommendation among users to the mining of users' potential preferences. Overall, the music recommendation algorithm's ability to make recommendations gets better and better [4].

Currently, searching online is the primary method of finding music. In other words, music labels—which frequently include song titles, singers, and musical genres—are used to search for songs [5]. Therefore, from the perspective of these conventional methods for retrieving music, they can only satisfy the need for a straightforward song search, and if the label is too small, they will not be able to effectively acquire music. The two most common methods of classifying music at the moment are manual classification and automatic music classification [6]. Manual classification refers to staff-by-staff classification of each piece of music. Manual classification methods are simple to use and have a respectable accuracy rate. Manual classification methods, on the other hand, place an undue emphasis on the musical expertise and interests of the staff, which results in inconsistent music classification standards and unstable classification outcomes. Big data, however, has created new opportunities and challenges for recommendation methods for massive amounts of music data [7]. The original recommendation algorithm needs to be updated in accordance with the complexity of processing massive amounts of data and the need to combine it with personalised user needs. On the other hand, urgent solutions are required for the problems with the original recommendation algorithm, such as the “cold start” issue with collaborative filtering recommendations. These types of musical elements are frequently found in songs because music labels are wealthy. Searching using only one label has significant limitations [8]. Additionally, it can be difficult to locate your preferred musical genre using only the song's title and associated label if you want to obtain music from a sizable library. Many people have started researching the automatic music style classification system in an effort to develop a more effective and precise system. The quantity of music available today is growing rapidly. The results of the manual classification method are still unstable and labor- and time-intensive. The modern society's demand for accurate and logical music classification cannot be fully satisfied by manual classification methods [9]. Automatic music classification methods are gradually replacing manual classification methods to enter people's musical worlds as computer science and technology, audio signal processing, machine learning, and other advance disciplines. On the other hand, new computer technologies like deep learning and big data processing emerge one after another. With more processing power and greater recommendation accuracy, these new technologies will aid in the development of new recommendation algorithms. The machine's computing power is constrained due to insufficient data consideration, and the training process takes too long. Therefore, human beings must set up every pattern that emerges during processing in advance if they want machines to make any kind of search classification. The rapid advancement of big data cloud storage and other technologies has made it possible for people to finally have enough data to support many of their questions, allowing for a clearer understanding of their core concerns and the creation of intricate models to address a variety of issues.

The innovations of this paper are as follows:

1. Machine learning is explained, and the means in this paper belongs to the category of machine learning. So it is necessary to make an introduction to the background. Artificial intelligence is the functions related to human intelligence performed by intelligent machines such as computers, including identification, judgment, proof, learning, and other thinking activities.
2. The neural network is explained. The means used in this paper is neural network, so it is necessary to introduce it. Artificial neural network was first put forward by foreign scientists, which can process message by imitating neurons.
3. Since I specifically use convolutional neural networks, it is important to understand them. A multilayer perceptron specifically created for two-dimensional image recognition is the convolutional neural network. It has some benefits that the conventional approach lacks, including strong fault tolerance, parallel processing, and self-learning capability. It can address issues with complex environmental messages, ambiguous background information, and illogical reasoning principles. It runs quickly and has good adaptive performance and a high resolution while allowing for large defects and distortions in the samples.

## 2. Related Work

Zhang suggested that music should be automatically classified based on the content of music signals, using autocorrelation coefficient, variance, mean value, and other features to represent music perception characteristics and using nearest neighbor algorithm as classifier [10]. Rosner suggested using the improved KNN algorithm to solve the multilabel classification problem of emotion [4]. Yang suggested that collaborative filtering should be combined with user context information, and the original user-data scoring model of collaborative filtering should be expanded to form a three-dimensional data model of user-data-context, and the correlation dimension should be expanded to achieve more accurate personalised recommendation [11]. Das suggested using 12-order mel-frequency cepstral coefficients MFCC (MFCC) and 1-order energy to represent music perception characteristics and using nearest neighbor algorithm as classifier [12]. Chen suggested to compare four multilabel classification algorithms. Through an experiment on a group of 593 samples, 30-second excerpts were extracted from them, and a group of labels were used to annotate them. The overall prediction results were basically satisfactory [13]. Sun suggested that third-party recommendations be used in mobile application scenarios. They use the current location of users as context information and collect preferences of other users at the current location as recommendations [14]. Kim suggested using new features such as harmonic coefficients in features and proposed a more robust music and speech classification algorithm [15]. Dorochowicz suggested the problem of combining user-generated labels with music content to classify artistic styles [16]. Nanni suggested a general architecture for context-aware recommendation system [17]. Wang suggested introducing wavelet transform into feature engineering and using neural network model in classification method [18]. López proposed a new language model and suggested the usefulness of clustering using tags and audio content. The findings demonstrate that tag features are superior to music content in terms of clustering artistic styles, and the proposed model can marginally enhance clustering performance by combining tags and music content [19]. Gerardo recommended using the Gaussian mixture model, which had good accuracy [20] for classifying musical genres. The multilabel classification problem was divided into numerous single-class problems, and Hsu suggested a two-dimensional method for categorising genres [21].

The processing of music has advanced quickly in recent years, and a lot of new music has been produced. People need to be able to quickly locate their favourite music as there is a lot of music available. A crucial component of multimedia applications is the classification of music genres. The amount of data on musical genres has grown significantly with the quick development of data storage, compression, and Internet technologies. Traditional manual retrieval methods are unable to meet peoples' needs for retrieval and classification of large music messages. The aforementioned issues will be resolved by the automatic classification of music by computers. Computer-aided music analysis is a brand-new interdisciplinary field whose research spans physics, signal processing, human-computer interaction, music theory, and music psychology, among other fields. The goal of this study is to examine this crucial factor.

## 3. Related Theories

### 3.1. Machine Learning

Machine learning, which is the core component of artificial intelligence, has always drawn people's attention as it has been applied more and more as science and technology have advanced. Learning is a crucial human skill, and as computers have advanced, they now have the capacity to learn things over time. The definition of artificial intelligence is the performance of tasks associated with human intelligence by intelligent machines like computers, including activities like identification, judgment, proof, learning, and other forms of thought. This illustrates the fundamental tenet and content of artificial intelligence, which is a branch of study into the rules governing human intelligence. The function of a function typically uses another function to process the input before receiving the output. The majority of machine learning has similar functions to functions, meaning that it has input and output, and the intermediate operation process requires our determination. In machine learning, we commonly refer to it as a model.

This paper provides a definition of big data based on ongoing research in the field: big data requires a new processing mode to have a significant amount of high-growth message assets, as well as stronger discovery and process optimization capabilities. Big data is clearly characterised by the four 4Vs: low value density, large data volume, diverse data types, and quick data processing. It used to be that the traditional data mining algorithm would use the data set to optimise the machine learning algorithm. However, the demand for data mining in the current large amount of heterogeneous data has proven challenging for this traditional machine learning method due to the current aspects of collection, retrieval, storage, sharing, analysis, and processing. Statistics, which was first applied in the processing and analysis of large amounts of data, is the foundation of data analysis. Machine learning, a subfield of artificial intelligence, aims to answer questions for particular objects through self-learning without programming. It can automate some functional operations and realise some aspects of human intelligence. The development of artificial intelligence technology began in the middle of the 20th century. It had a significant impact on society's overall development in addition to facilitating people's ability to produce and live more conveniently.

In the summer of 1956, the concept of “artificial intelligence” was first put forward. Artificial intelligence began to develop rapidly after the advent of computers because people really have tools that can simulate human thinking. Nowadays, artificial intelligence is no longer a niche research topic. Almost all universities of science and engineering in the world are studying this subject and even set up special research institutions for it. More and more undergraduate or graduate students majoring in computer, automatic control, and software engineering take artificial intelligence as their research direction. There are a number of definitions for big data, but generally speaking, it refers to a very large-scale data processor with capabilities for data acquisition, storage, management, and analysis.

Big data must be analysed and sorted by distributed architecture because, technically speaking, it cannot be processed by a single computer. Additionally, this enables it to gather vast amounts of data in a distributed manner. In order for big data to effectively accommodate the retention of massive amounts of data, special techniques must be used in its development. Studying the machine learning algorithm in a big data environment, that is, using machine learning to mine the priceless knowledge points already present in the current dynamic complex database, is of great practical importance. Artificial intelligence, machine learning, and big data analysis are closely related, and the corresponding fields are capable of realising their unique functions. In the real world, similar questions are resolved in various fields using big data processing and analysis, along with artificial intelligence and machine learning techniques.

### 3.2. Neural Network

Computer data is growing alarmingly quickly as a result of the use of digital equipment and the advancement of sensor technology. In the field of machine learning, the challenge of processing and analysing large amounts of data is a hot topic. With the explosion of big data comes the emergence of data science, an interdisciplinary field. Designing and creating algorithms that can intelligently “learn” from actual data is the primary goal of machine learning research. These algorithms can automatically discover patterns and rules that are hidden in data. The idea of an artificial neural network, which processes messages by resembling neurons, was first advanced by scientists from outside the country. Artificial intelligence technology has continuously advanced alongside the development of social science and technology. Artificial intelligence machines can issue corresponding instructions in accordance with people's design requirements, mimic human behaviour, have specific induction, and issue corresponding instructions in accordance with human behaviour to produce corresponding results with the development of computer Internet. A learning network with several hidden layers on top of a neural network is known as “deep learning.” Along with the rise of the message age, deep learning was born. Numerous neurons connected by programmable connection weights make up an artificial neural network.

Artificial neural networks have excellent self-organization and self-adaptability as well as strong learning capabilities. They also have large-scale parallel processing and distributed information storage. After a protracted period of development, artificial neural networks have recently made ground-breaking strides in their research and have seen widespread use in a variety of fields. Machine learning techniques such as deep neural network theory are based on how the human brain learns. The term “deep learning” is another name for it. The fundamental concept of a deep neural network can be summed up as follows: unsupervised learning is used to pretrain each network layer, followed by gradual layer training, input from one layer being used as the output for the next, and supervised learning is used to fine-tune all learning layers. The use of artificial intelligence techniques can increase the capabilities of machines and support the continued development of identification techniques for artificial intelligence.

On the basis of neural network algorithm, modern technique is continuously integrated, and message collection, storage, analysis, and application are realized by using the cross interaction between neurons, so as to improve the recognition sensitivity and resolution efficiency of artificial intelligence recognition technique, promote the in-depth integration of neural network algorithm in the field of intelligent recognition, and expand the application scope of artificial intelligence recognition technique. Deep neural network is a kind of neural network with multiple hidden layers, which has a specific structure and training mode. Its idea comes from the hierarchical processing mechanism of human brain to visual message. From the original data, it can automatically learn effective feature expressions through multilayer structure and realise classification and recognition at the output layer. The classical neural network model is shown in Figure 1.

Deep neural networks differ from traditional neural networks primarily due to the training mechanism. Deep neural networks pretrain primarily layer by layer in the training mechanism in order to overcome the drawbacks of traditional neural networks, such as slow training speed and easy overfitting. The neural network algorithm has received attention and has been heavily utilised in the field of artificial intelligence as a result of the development of cloud computing and big data techniques in recent years. Logic, computer science, and many other disciplines are all integrated by deep neural networks. They encourage the development of artificial intelligence methods that can think and act like people, learn like people, and enhance their capacity to perceive and react to their environment. The algorithm and the choice of algorithm parameters directly affect whether the neural network algorithm can achieve global convergence and convergence speed, but most algorithms currently cannot provide the formula for parameter selection.

## 4. Music Classification Based on Feature Extraction and Neural Network

### 4.1. Convolutional Neural Network

With the advent of artificial intelligence era, people's requirements for target recognition and detection are further improved. The performance of traditional machine learning algorithms cannot meet people's needs. Convolutional neural network (CNN) has shown a good effect in handwritten numeral recognition in the early days. Because of the limitation of memory and hardware at that time, a large amount of training data could not be obtained, which made the network unable to expand larger images, resulting in a decrease of research heat at that time. Specifically created for identifying two-dimensional images, convolutional neural networks are multilayer perceptrons. It has some benefits that the conventional technique does not, including strong fault tolerance, parallel processing, and self-learnability. It is capable of addressing issues like complex environmental messages, hazy background information, and murky reasoning principles. It runs quickly, exhibits good adaptive performance, and has a high resolution while allowing for significant distortions and defects in the samples. A learning model from beginning to end is provided by convolutional neural networks. Traditional gradient descent techniques can be used to train the model's parameters. Convolutional neural networks that have been trained can extract and classify an image's features, as well as learn their characteristics.

Let the *D*2-layer output vector *h*_2_ be (*x*_1_, *x*_2_,…, *x*_*N*_) and let *σ*_2_ and *μ*_*h*_′ be the network training parameters; then, the *BN*-layer calculation process can be expressed as

(1) $$\begin{array}{c} \text{BN}\left(x_{1},x_{2},\ldots ,x_{N}\right)=\left(\frac{\left(x_{1}-\mu_{h}\right)\sigma_{2}}{\sigma_{1}+\mu_{h}^{\prime }},\frac{\left(x_{2}-\mu_{h}\right)\sigma_{2}}{\sigma_{1}+\mu_{h}^{\prime }},\ldots ,\frac{\left(x_{N}-\mu_{h}\right)\sigma_{2}}{\sigma_{1}+\mu_{h}^{\prime }}\right). \end{array}$$

Let the input vector of *Soft*max be (*y*_1_, *y*_2_,…, *y*_*M*_); then,

(2) $$\begin{array}{c} \text{Soft}\max\left(y_{1},y_{2},\ldots ,y_{M}\right)={\left[\sum_{i=1}^{M}\exp\left(y_{i}\right)\right]}^{-1}\left(\exp\left(y_{1}\right),\;\exp\left(y_{2}\right),\ldots ,\;\exp\left(y_{M}\right)\right). \end{array}$$

The neural network layer is

(3) $$\begin{array}{c} h_{1}=\text{Relu}\left(aW_{1}+b_{1}\right),\\ h_{2}=\text{Relu}\left(h_{1}W_{2}+b_{2}\right),\\ \mu_{h}^{\prime }=\text{BN}\left(h_{2}\right),\\ \text{out}=\text{Soft}\max\left(\mu_{h}^{\prime }W_{3}+b_{3}\right). \end{array}$$

Convolutional neural networks have advanced quickly since the early twenty-first century as a result of the development of deep learning theory and the advancement of numerical computing technology. Convolutional neural networks have the advantage over conventional methods in that they can automatically extract target features, find feature rules in sample sets, and address the problems associated with the low efficiency and low classification accuracy of manual feature extraction. Because of this, convolutional neural networks are widely used in image classification, target recognition, natural language processing, and other fields and have achieved remarkable results. Despite being surrounded by a lot of data, humans can always find a clever way to receive the information they need. The central problem of pattern recognition theory research has always been how to efficiently and accurately mimic the human brain's ability to extract the most important information from a large amount of perceptual data.

Every level adds the weight determined by a set of weights to the input, which is taken from a local area of the previous level at each level. The output of the previous level is said to have been convolved with a kernel function to produce the current level, thus, the name convolutional neural network. Convolutional neural networks are a significant area of research in the field of neural networks. They have the property that the local area of the top layer, via the convolution kernel with shared weights, excites the features of each layer. Convolution neural networks are better suited for learning and expressing features than other neural network techniques because of this characteristic.

Let the input of the convolutional neural network be the original image (*X*_0_, *Y*_0_) and use *X*_*i*_ to represent the characteristic map of the *i* rd layer of the convolutional neural network, and you can get

(4) $$\begin{array}{c} X_{i}=F\left(X_{i-1}*W_{i}+b_{1}\right). \end{array}$$

Downsampling the characteristic map is as follows:

(5) $$\begin{array}{c} X_{i}=\text{Subsampling}\left(X_{i-1}\right). \end{array}$$

The network execution output is

(6) $$\begin{array}{c} O_{p}=F_{n}\left(\ldots \left(F_{2}\left(F_{1}\left(X_{0}W_{1}+b_{1}\right)W_{2}+b_{2}\right)\ldots \right)W_{n}+b_{n}\right). \end{array}$$

The learning rate parameter *η* is used to control the strength of residual back propagation:

(7) $$\begin{array}{c} E\left(W,b\right)=L\left(W,b\right)\frac{\lambda }{2}W^{T}W,\\ W_{i}=W_{i-1}-\eta \frac{\partial E\left(W,b\right)}{\partial W_{i-1}},\\ b_{i}=b_{i-1}-\eta \frac{\partial E\left(W,b\right)}{\partial b_{i-1}}. \end{array}$$

The nonlinear function is

(8) $$\begin{array}{c} f\left(x\right)=\frac{1}{1-e^{-x}}. \end{array}$$

*W*_*i*_ denotes the weight vector of the convolution kernel of the *i* nd layer. The operation symbol “*∗*” represents the convolution operation between the convolution kernel and the *i* − 1 rd layer image or the feature map.

A convolutional neural network can be thought of as a special type of multilayer perceptron or feedforward neural network with local connections and weight sharing, in which a lot of neurons are arranged in a specific way to respond to overlapping regions of the visual field. Convolutional neural networks have recently undergone significant advancement thanks to the research and development carried out by numerous top academics from both home and abroad. In some tasks, their level of recognition has even reached or surpassed that of humans. Convolutional neural network has produced many ground-breaking accomplishments and outcomes in computer vision in recent years. Convolutional neural networks have gained significant attention throughout the field due to their strong feature learning and classification capabilities, and more and more researchers are realising their value for analysis and research.

### 4.2. Model Construction

This model involves creating a website where users can upload music. The audio data will then be moved to the background of the page for analysis. Additionally, the likelihood of the current music's genre can be seen in real time by clicking the audio page to start playing. The music spectrum is classified using the CNN classification model, and the fundamental feature vectors are obtained. A more precise piano music feature library can be created by optimising the feature vectors of the music. Music similarity and user preference features can both be computed using a feature library.  Figure 2 displays the CNN training procedure.

Since 2012, researchers have used the Alexnet network model in the competition to surpass the previous best record and have won the title with a clear advantage. This has established the convolutional neural network as the foundational technology in computer vision. Since then, convolutional neural networks have gained widespread acceptance in both academia and industry, and an increasing number of researchers have committed their careers to studying them. In the fields of speech segmentation, image segmentation, and image classification, among other research areas, convolutional neural networks have achieved great success. Convolution neural networks have, however, received relatively little study in the areas of music classification and recognition. This paper's research on this crucial topic is its main body. The gradient change rhythm of the algorithm in this paper is better than that of the traditional algorithm, as can be seen from Figures 3–6. This is because the larger learning rate causes the larger gradient change.

The front-end interactive interface, in order to increase the user experience, has the audio upload function in the front-end page, which allows users to upload music, so as to show the background. In order to further increase the visualization effect, the front page can play the uploaded music. During the playing process, the page will show the probability of the current music in real time. After the playing, it will show the probability of each genre of the current music. The classification of the front desk will change with the increase of audio playing time. If the user's favorite music already exists in the music library, you can directly look up the feature library. If it does not exist, we need to generate spectrum samples and use CNN classification model to predict and classify, and get feature vectors. In the first layers of the model of convolution neural network of auditory characteristics, the features are learned continuously through the cooperation and accumulation of convolution operation, pooling operation, and activation function, and the task of extracting higher-level features from time-frequency feature coefficients is completed, which is convenient for subsequent classification. From Tables 1 and 2 and Figures 7 and 8, it can be seen that this algorithm is 12% better than the traditional algorithm, and its ability is strong at the same number of iterations.

In the later layers of the model of convolutional neural network of auditory characteristics, the importance of each learned feature is calculated through the full connection layer, so that music can be better classified. The trained neural network has been saved on the server, and when the music is uploaded, the concert will automatically analyze the music genre from the background. For instance, the experiment chose a piece of music from the classical music genre. The system recognised the song as belonging to the appropriate genre after I uploaded it to a reliable website I had created. Neural network predictions are generally accurate, and the majority of them can be seen. The music is of the classical genre. The time-frequency features of music are divided into N regions. Compared with general convolutional neural networks, convolution kernels of convolutional neural networks based on auditory characteristics are no longer globally shared, so that convolution kernels in various frequency regions can learn the required features of their respective frequency regions, overcoming the disadvantage that general convolutional neural networks consistently treat each frequency domain feature in time-frequency features and ignore the difference of frequency domain message. Compared with general convolutional neural networks, convolutional neural networks based on auditory characteristics in music classification tasks are more in line with auditory characteristics.

## 5. Conclusions

With the rapid development of Internet and multimedia message technique, the number of music is exploding, and people can choose more and more music. Only by properly classifying the massive music resources and establishing an efficient music retrieval system can people accurately and quickly search for their desired music according to various preferences and needs. With the development of artificial intelligence technique, the concept of deep learning has gradually been applied to all aspects of research, and neural networks have gradually replaced traditional feature extraction and other steps. For example, the current convolutional neural networks have been applied to music, images, texts, and other fields. Traditional music classification means rely on manual labelling to classify music. Nowadays, in the era of big data where the number of music is exploding, it is obviously inefficient and unrealistic to complete the task of classifying massive music by manual labelling. This is the research in this field. From this research, it is concluded that this algorithm is 12% better than the traditional algorithm. At the same number of iterations, it has strong ability and is suitable for being widely put into practice.

## Figures and Tables

**Figure 1:** Classical neural network model.

**Figure 2:** CNN training process.

**Figure 3:** Microcosmic score of various time analysis windows.

**Figure 4:** Macro score of various time analysis windows.

**Figure 5:** Accuracy comparison.

**Figure 6:** Comparison of gradient changes.

**Figure 7:** Comparison of network training.

**Figure 8:** ROC curve of network model.

**Table 1:** Comparison of network training.

	0	25	50	75	100	125	150	175	200	225	250
Algorithm	1347	1529	1146	1783	1655	1494	1366	1483	1296	1588	1799
Traditional algorithm	1479	1396	1578	1364	1139	1297	1345	1635	1524	1255	1397

**Table 2:** ROC curve of network model.

	0	0.025	0.05	0.075	0.1	0.125	0.15	0.175	0.2	0.225	0.25
Algorithm	0.84	0.79	0.81	0.85	0.74	0.83	0.93	0.90	0.92	0.87	0.89
Traditional algorithm	0.74	0.83	0.85	0.75	0.78	0.71	0.76	0.84	0.75	0.81	0.77

## Data Availability

The data used to support the findings of this study are available from the corresponding author upon request.
